The article "Two novel Mg(II)-based and Zn(II)-based complexes: inhibiting growth of human liver cancer cells" was published in 2017. Journal: Braz J Med Biol Res.

# Two novel Mg(II)-based and Zn(II)-based complexes: inhibiting growth of human liver cancer cells

**DOI:** 10.1590/1414-431X20176929

**Published:** 2017-12-18

**Authors:** N. Liu, D. Ding, L. Wang, H. Zhao, L. Zhu, X. Geng

**Affiliations:** 1 Department of Critical Care Medicine, The First Affiliated Hospital of Anhui Medical University, Hefei, Anhui, China; 2 Department of Physiology, Anhui Medical College, Hefei, Anhui, China; 3 Department of Physiology, Basic Medical College of Anhui Medical University, Hefei, Anhui, China; 4 Department of General Surgery, The First Affiliated Hospital of Anhui Medical University, Hefei, Anhui, China

**Keywords:** Coordination polymer, Pillar-layered, Liver cancer

## Abstract

Two new Mg(II)-based and Zn(II)-based coordination polymers, {[Mg_3_(BTB)(DMA)_4_](DMA)_2_}_n_ (**1**, H_3_BTB=1,3,5-benzenetrisbenzoic acid, DMA=N,N-dimethylacetamide) and {(H_2_NMe_2_)_2_[Zn_3_(BTB)_2_(OH)(Im)](DMF)_9_(MeOH)_7_}_n_ (**2**, Im=imidazole, DMF=N,N-dimethylformamide), have been successfully synthesized and structurally characterized under solvothermal conditions. **1** contains a linear [Mg_3_(COO)_6_] cluster that connected by the fully deprotonated BTB^3-^ ligands to give a ***kgd***-type 2D bilayer structure; **2** represents a microporous 3D pillar-layered system based on the binuclear Zn units and pillared Im ligands, which shows a (3,5)-connected **hms** topological net. In addition, *in vitro* anticancer activities of compounds **1** and **2** on 4 human liver cancer cells (HB611, HHCC, BEL-7405 and SMMC-7721) were determined.

## Introduction

Cancer is presently responsible for about 25% of deaths in developed countries and for 15% of all deaths worldwide (1). It is therefore considered one of the foremost health problems, with about 1.45 million new cancer cases expected yearly (2,3). Antitumor chemotherapy is a very active field of research, and a large amount of information on the topic is generated every year (4,5). However, there is a clear need for new treatments, from the medicinal chemistry and drug design point of view (6).

In recent years, aromatic multi-carboxylate acid compounds have been widely used as versatile ligands involved in various metal chelation reactions to form transition metal complexes with interesting properties in material sciences and biological systems (7,8). These complexes can be easily synthesized from simple starting materials, where the metal ions, ligands, and coordination modes are the important factors for the self-assembly processes (9,10). 1,3,5-benzenetrisbenzoic acid is a versatile ligand, which acts as monodentate or bridging group with end-on or end-to-end coordination mode to form complexes with interesting structures.

In this work, two new ***kgd***-type 2D bilayer and pillar-layered coordination polymers, namely {[Mg_3_(BTB)(DMA)_4_](DMA)_2_}_n_ (**1**) and {(H_2_NMe_2_)_2_[Zn_3_(BTB)_2_(OH)(Im)](DMF)_9_(MeOH)_7_}_n_ (**2**), were obtained (Figure 1) and their anticancer activity was evaluated.

**Figure 1.** Schematic representation of the H_3_BTB and Im ligands used in this research.

## Material and Methods

### Apparatus and materials

All starting materials and reagents used in this research were obtained commercially and used without further purification. To obtain infra-red (IR) spectra (400∼4000 cm^-1^), we used a Brucker Equinox-55 spectrophotometer (Bruker, Germany). Element analyses (C, H, and N) were determined with a Vairo EL III analyzer (Elementar, Germany). Single crystal X-ray diffraction was carried out by an Oxford Xcalibur E diffractometer (Bruker Optics, Germany). A XT-4 micro melting apparatus (Ledon, China) was used to determine the melting points, and the thermometer remained uncorrected.

### Synthesis and characterization of complexes 1 and 2

A mixture of Mg(NO_3_)_2_·6H_2_O (25.6 mg, 0.1 mmol), H_3_BTB (24.3 mg, 0.05 mmol), and DMA/H_2_O/CH_3_CN (V/V/V = 2/1/1, 5 mL) was sealed in a Teflon-lined stainless-steel vessel (20 mL), and heated to 120°C in 12 h, kept at 120°C for 3 days then slowly cooled to room temperature in 24 h. The colorless block crystals were collected, washed with DMF, and air dried. Details are as follows: Yield: 25.3 mg, 36% (based on H_3_BTB ligand). Mp. >300°C. IR (KBr pellets) cm^-1^: 3440 (w), 2933 (w), 2433 (w), 1652 (w), 1103 (w), 930 (s), 810 (w), 682 (w), 597 (m). Elemental analysis for the framework of **1** (C_51_H_69_Mg_3_N_6_O_12_) was: C=59.23; H=6.44; N=8.29%. Calculated: C=59.41; H=6.75; N=8.15%.

A mixture of Zn(NO_3_)_2_·6H_2_O (0.1 mmol, 0.031 g), H_3_BTB (10 mg, 2.2 mmol) and imidazole (4.65 mg, 6.6 mmol) was added to a solution of MeOH (1 mL), H_2_O (2 mL), and DMF (2.5 mL) in a 25 mL Teflon-lined stainless steel container. The container was heated at 120°C for 48 h, and then cooled to room temperature at 2°C/min. The resulting material, in the form of light yellow single crystals, was washed with MeOH and left to air dry. Details are as follows: Mp. >300°C. IR (KBr pellets) cm^-1^: 3134 (w), 2911 (w), 2410 (w), 1732 (w), 1143 (w), 976 (s), 808 (w), 689 (w), 590 (m). Analytical results found for compound **2** (C_137_H_178_N_21_O_36_Zn_6_) were: C=53.45; H=5.44; N=9.21%. Calculated: C=53.30; H=5.81; N=9.53%.

### Crystal structure determination

Suitable single crystals of compounds **1** and **2** were carefully selected under optical microscope and glued on thin glass fibers. The intensity data of **1** and **2** was obtained on an Oxford Xcalibur E diffractometer. The empirical absorption corrections were applied to the data using the SADABS system. This structure was solved by direct method and refined by full-matrix least-squares method on *F* ^2^ using the SHELXS–97 program (11). All non-hydrogen atoms of **1** and **2** were refined anisotropically, and all the hydrogen atoms attached to carbon atoms were fixed at their ideal positions. Pertinent crystal data and structural refinement results for compounds **1** and **2** are summarized in Table 1.

**Table 1.** Crystal data and structure refinements for compounds **1** and **2.**

	1	2
Formula	C_19.50_H_21_Mg_0.75_N_1.50_O_4.5_	C_99_H_71_N_10_O_20_Zn_6_
*M*r	366.61	2112.87
Temperature/K	293 (2)	293 (2)
Crystal system	Monoclinic	Monoclinic
Space group	*P*2_1_/*n*	*P*2_1_/*c*
*a*/Å	12.4947 (4)	24.3437 (8)
*b*/Å	25.7603 (9)	28.0222 (6)
*c*/Å	13.7797 (5)	19.8450 (4)
*α*/°	90	90
*β*/°	99.622 (3)	102.182 (3)
*γ*/°	90	90
*V*/Å^3^	4372.8 (3)	13232.7 (6)
*Z*	8	4
*D*_calc_/g·cm^-3^	1.114	1.061
*μ*(Mo Kα)/mm^-1^	0.098	1.647
*θ* range/°	2.999 to 24.999	3.594 to 73.853
Reflections collected	15554	52557
No. unique data [*R*(int)]	7224 [0.0347]	26073 [0.0249]
No. data with *I* ≥ 2*σ*(*I*)	4924	21300
*R*_1_	0.0681	0.0430
*ωR*_2_(all data)	0.1939	0.1320
CCDC	1561061	1561062

### Antitumor activity

Four human liver cancer cells (HB611, HHCC, BEL-7405 and SMMC-7721) were grown in a RPMI 1460 medium supplemented with 10% fetal calf serum, 100 μg/mL penicillin and 100 μg/mL streptomycin. Cells were incubated at the temperature of 37°C in a moist incubator with 95% air and 5% CO_2_. Cells at exponential growth were diluted to 5×10^4^ cells/mL with RPMI1640, and then seeded on 96-well plates at a volume of 100 μL per well, and incubated for 24 h at 37°C in 5% CO_2_. After incubation of cells for up to 96 h, the medium was removed from each cell and 150 μL of MTT (0.5 mg/mL) solution, diluted 10-fold by RPMI 1460 was subsequently added. The IC_50_ values were measured by depicting the ratio viability versus concentration on a logarithmic chart and obtaining the concentration where 50% of cells were inhibited. In order to get mean values, each experiment was conducted at least three times in the same way.

## Results and Discussion

### Molecular structure

As shown in Figure 2A, the asymmetric unit of **1** contains two crystallographically independent Mg(II) with 1/2 (Mg1) and 1 (Mg2) occupancies, one BTB^3-^ ligand, two coordinated DMA and one lattice DMA molecule. Both Mg1 and Mg2 reveal similar six-coordinated octahedral geometries. Mg1 is located at an inversion center of (-1/2, 0, 1/2) and surrounded by six carboxylate O atoms from six different BTB ligands with the Mg–O lengths ranging from 2.021(2) to 2.037(2) Å. Mg2 is coordinated by four carboxylate O atoms from three BTB^3-^ ligands and two O atoms from two coordinated DMA molecules with the Mg–O lengths in the range of 2.031(2)–2.203(3) Å. With the aid of a bridged carboxylate, two symmetry-related Mg2 ions and one Mg1 ion are held together to generate a [Mg_3_(COO)_6_] congregation (Figure 2B). Due to the restriction of the terminal solvent molecules of Mg2, only a discrete [Mg_3_(COO)_6_] subunit is achieved. These trimeric clusters are further extended by BTB^3-^ ligands along the *ab* plane to give a 2D bilayer pattern (Figure 2C). The Mg2⋯Mg2 distance in the linearly arranged Mg_3_ array is about 7.199 (2) Å, which is long enough to accommodate the bilayer network. These 2D bilayers adopt a parallel stacking arrangement to afford a 3D supramolecular architecture without classic H-bonding or pi-pi interaction. Topologically, the Mg_3_ SBUs and BTB ligands can be regarded as 6- and 3-connected nodes, respectively, and afford a binodal (3,6)-connected ***kgd*** network with the point symbol of {4^3^}_2_{4^6^·6^6^·8^3^} (Figure 2D).

**Figure 2.** *A*, View of the asymmetric unit of **1**; *B*, view of the [Mg_3_(COO)_6_] subunit of **1** (symmetry code A: 2-X, 1-Y, 2-Z); *C*, view of the 2D bi-layered structure of **1**; *D*, the binodal (3, 6)-connected ***kgd*** network for **1**.

The structural analysis results indicate that compound **2** crystallizes in the monoclinic space group P2_1_/c, and shows a 2-fold interpenetrated network. The asymmetric unit of **2** consists of six Zn(II) ions, three BTB^3^-ligands, five deprotonated Im ligands, two coordinated DMF molecules, and two lattice disordered H_2_NMe_2_ cations. The six Zn(II) ions exhibit two different coordinating modes (Figure 3A): Zn1, Zn2, Zn4 and Zn5 atoms are four-coordinated by three O atoms from three different carboxylic acid groups on the BTB^3-^ ligands and one N atom from the deprotonated Im ligand, forming a distorted tetrahedral coordination mode; atoms Zn3 and Zn6 are five-connected by one(two) N atom(s) from the Im ligand(s) and three(two) O atoms from the carboxylic acid groups, resulting in a pyrometric geometry. Zn1-Zn6, Zn2-Zn3 and Zn4-Zn5 atoms are linked by the carboxylic groups to afford the binuclear Zn secondary building units (SBUs), which are joined by the Im pillars along the *c* axis to give rise to the 1D SBU chains (Figure 3B). In addition, the BTB^3-^ ligand links with the binuclear Zn SBUs along *bc* plane to give the 6^3^ layer, and the Im ligands act as pillars between 2D sheets to form the three-dimensional (3D) framework. Due to its large solvent-accessible volume, such a framework might be large enough to accommodate another identical one to be interpenetrated, thus forming a doubly interpenetrated 3D framework with one-dimensional (1D) channel (Figure 3C). Notably, the 1D channels are decorated with Im groups, which might be favorable for the formation of a H-bond interaction. The calculated void space per unit cell for guest-free framework is 40% as revealed by the PLATON analysis [probe radius: 1.4 Å]. From the topological point of view, the 3D structure of **2** can be rationalized as a 2-fold interpenetrated **hms**-type (3,5)-connected network by considering the BTB^3-^ ligand, binuclear Zn unit and the Im pillar as a 3, 5 and 2-connected node. (Figure 3D).

**Figure 3.** *A*, View of the coordination modes of Zn(II) ions in **2**; *B*, view of 1D secondary building unit chains and the 3D pillared framework; *C*, view of the 2-fold interpenetrated 3D framework of **2**; *D*, the **hms**-type (3,5)-connected topology for **2.**

### Anticancer activity

The cytotoxicity of the title compounds **1** and **2**, reference drug carboplatin, organic ligands H_3_BTB and Im against HB611, HHCC, BEL-7405 and SMMC-7721 cell lines were evaluated by MTT assay, and the IC_50_ values derived from the experimental data are shown in Table 2. The two organic ligands were ineffective against all cell lines (IC_50_ >100 μM). At this concentration, H_3_BTB and Im would exert high cytotoxicity against normal cells, thus we conclude that it did not exert inactivation towards these cell lines.

**Table 2.** Growth inhibitory effects of **1**, **2**, carboplatin, H_3_BTB and Im on HB611, HHCC, BEL-7405 and SMMC-7721 cancer cells.

Compounds	IC_50_ (μM)			
	HB611	HHCC	BEL-7405	SMMC-7721
H_3_BTB	>100	>100	>100	>100
Im	>100	>100	>100	>100
**1**	20	25	30	32
**2**	26	23	27	35
Carboplatin	25	30	25	40

However, after the cancer cells were incubated in the presence of compounds **1** and **2** for 72 h, the IC_50_ values for the compound ranged from 20 to 35 μM, which is similar or even lower than that of carboplatin (25–40 μM), indicating that the title compounds **1** and **2** exhibited anticancer activity against these cell lines in different degrees.

According to the above-mentioned data, it can be concluded that compared with organic ligands H_3_BTB and Im, the anticancer activity of compounds **1** and **2** was more effective. However, additional studies are needed to define the mechanism underlying the antitumor activity of these compounds and evaluate their efficacy *in vivo*.
